RETRACTED

# Metal tolerance protein MTP6 affects mitochondrial iron and manganese homeostasis in cucumber

**DOI:** 10.1093/jxb/ery342

**Published:** 2018-10-09

**Authors:** Magdalena Migocka, Ewa Maciaszczyk-Dziubinska, Karolina Małas, Ewelina Posyniak, Arnold Garbiec

**Affiliations:** 1 University of Wroclaw, Institute of Experimental Biology, Department of Plant Molecular Physiology, Kanonia, Wroclaw, Poland; 2 University of Wroclaw, Institute of Experimental Biology, Department of Genetics and Cell Physiology, Kanonia, Wroclaw, Poland; 3 University of Wroclaw, Institute of Experimental Biology, Department of Animal Developmental Biology, Sienkiewicza, Wroclaw, Poland

**Keywords:** CDF (cation diffusion facilitator) family, *Cucumis sativus*, iron, manganese, mitochondria, MTP (metal tolerance protein) family

## Abstract

Members of the cation diffusion facilitator (CDF) family have been identified in all kingdoms of life. They have been divided into three subgroups, namely Zn-CDF, Fe/Zn-CDF, and Mn-CDF, based on their putative specificity to transported metal ions. The plant metal tolerance protein 6 (MTP6) proteins fall into the Fe/Zn-CDF subgroup; however, their function in iron/zinc transport has not yet been confirmed. Here, we characterized the MTP6 protein from cucumber, *Cucumis sativus*. When expressed in yeast and in protoplasts isolated from Arabidopsis cells, CsMTP6 localized in mitochondria and contributed to the efflux of Fe and Mn from these organelles. Immunolocalization of CsMTP6 in cucumber membranes confirmed this association with mitochondria. Root expression and protein levels of CsMTP6 were significantly up-regulated in conditions of Fe deficiency and excess, but were not affected by Mn availability. These results indicate that MTP6 proteins contribute to the distribution of Fe and Mn between the cytosol and mitochondria of plant cells, and are regulated by Fe to maintain mitochondrial and cytosolic iron homeostasis under varying conditions of Fe availability.

## Teaser

CsMTP6 contributes to the distribution of Fe and Mn between the cytosol and mitochondria of cells, and is regulated by Fe to maintain mitochondrial and cytosolic iron homeostasis.

## Introduction

Iron plays an essential role in many housekeeping cellular functions, including respiration, photosynthesis, Fe-S cluster assembly, and heme synthesis, but it can also be highly reactive and toxic as a catalyst of the Fenton reaction when present in excess (Winterbourn, 1995; Briat *et al.*, 2010). The maintenance of iron homeostasis is particularly relevant for plants, which can find themselves exposed to different Fe regimes and which require continuous Fe delivery for chlorophyll synthesis and photosynthetic reactions. The rate of Fe uptake and storage in plants is also important for human nutrition, since it may significantly affect the yield and nutritional value of crops. Hence, a more comprehensive understanding of the molecular mechanisms that regulate plant iron homeostasis would be beneficial for the breeding or engineering of crops that are enriched in Fe and more tolerant of Fe-deficient soils.

RETRACTED

Over the last decade, the molecular mechanisms underlying Fe acquisition and uptake by plants have been identified. They include the key genes involved in two different strategies of iron uptake: the reduction strategy used by dicotyledonous and non-graminaceous monocotyledonous species (strategy I), and the chelation strategy used by graminaceous species (strategy II). Iron-uptake strategy I involves genes encoding plasma membrane Fe^3+^-chelate reductase FRO2 and the Fe^2+^ transporter IRT1 (iron-regulated transporter 1), which are involved in the reduction of soil Fe^3+^ to Fe^2+^ followed by the transport of ferrous ions into the root cells (Eide *et al.*, 1996; Robinson *et al.*, 1999; Vert *et al.*, 2002). The genes involved in iron-uptake strategy II encode proteins involved in the synthesis and secretion of hexadentate Fe^3+^-chelating compounds (phytosiderophores, mugineic acid) and the specific plasma membrane Fe^3+^-phytosiderophore importer YS1 (yellow stripe 1) (Curie *et al.*, 2001). Members of the YSL (yellow stripe-like) family are also involved in the long-distance transport between different plant tissues and organs (Curie *et al.*, 2009).

In contrast to iron uptake, the partitioning of Fe between organelles in plant cells and the regulation of this process are less well understood. The regulation of intracellular compartmentation of Fe is likely to determine the level of storage and tolerance. A few proteins involved in Fe transport across the vacuolar membrane have already been identified, and these include VIT1 (vacuolar iron transporter) and the MTP8 (metal tolerance protein 8) transporter, which are involved in the loading of iron into the vacuole, and the natural resistance-associated macrophage proteins NRAMP3 and NRAMP4, which release Fe from the vacuoles in response to deficiency (Thomine *et al.*, 2003; Lanquar *et al.*, 2005; Kim *et al.*, 2006; Chu *et al.*, 2017; Eroglu *et al.*, 2017). It has been shown in Arabidopsis that all these four proteins play important roles during embryo development and seed germination. VIT1 is expressed in the endodermal cells surrounding the embryonic vasculature, whereas MTP8 localizes in the hypocotyl cortex cells and sub-epidermal cells of the embryonic cotyledons (Kim *et al.*, 2006; Chu *et al.*, 2017; Eroglu *et al.*, 2017). Both proteins are able to transport Mn in addition to Fe; however, VIT1 is primarily responsible for the storage of Fe in seeds, whilst MTP8 determines the pattern of seed Mn distribution (Kim *et al.*, 2006; Chu *et al.*, 2017; Eroglu *et al.*, 2017). Nevertheless, phenotypic analyses of Arabidopsis *vit1*, *mtp8*, and *vit1mtp8* loss-of-function mutants has shown that VIT1 can substitute for MTP8 when the latter is not functional, and vice versa (Chu *et al.*, 2017; Eroglu *et al.*, 2017). In addition, MTP8 is important for Mn stress tolerance and contributes in the detoxification of Mn under Fe-deficiency conditions (Eroglu *et al.*, 2016; Chu *et al.*, 2017). Similar to VIT1 and MTP8, the NRAMP3 and NRAMP4 proteins from Arabidopsis are also able to transport Fe and Mn, and both have been shown to be required for the release of Fe and Mn from the vacuoles of germinating seeds and mature leaves, respectively (Lanquar *et al.*, 2005, 2010). In seeds, NRAMP3 and NRAMP4 are expressed in the endodermal cells of the embryo, similarly to VIT1 (Lanquar *et al.*, 2005; Kim *et al.*, 2006). These three proteins are thought to form a functional module responsible for the vacuolar accumulation of Fe during embryo development and the efficient remobilization of Fe during seed germination (Mary *et al.*, 2015). The activity of this module is critical for the proper growth and development of seedlings under Fe deficiency (Lanquar *et al.*, 2005; Kim *et al.*, 2006). As VIT1, NRAMP3, and NRAMP4 transport Mn, this model may also function in the efficient vacuolar storage and remobilization of Mn in the endodermal cells of Arabidopsis embryos.

RETRACTED

Apart from the vacuole, the central roles in the cellular Fe economy of plants are played by plastids and mitochondria, which house the crucial processes of Fe metabolism, including heme biosynthesis, Fe-S cluster assembly, and Fe storage (Jain and Connolly, 2013). As integral parts of electron transfer chains, the Fe-containing compounds are essential for chloroplast photosynthesis and mitochondrial respiration, the major cellular pathways for energy conversion. However, despite its importance, Fe can also be highly reactive and toxic when it accumulates to high levels within the mitochondria and plastids of plant cells. Iron overload has long been associated with oxidative stress, which results from the Fe-catalysed formation of hydroxyl radicals that can damage DNA and proteins (Halliwell *et al.*, 1992). Thus, the Fe content in the mitochondria and plastids must be carefully regulated to ensure an adequate supply while avoiding its over-accumulation to toxic levels.

RETRACTED

The molecular mechanisms underlying the transport of Fe in and out of plastids and mitochondria have not yet been fully elucidated. Proteins involved in Fe loading into plant mitochondria and plastids have been recently discovered in rice (*Oryza sativa*) and Arabidopsis. The rice mitochondrial iron transporter (MIT) belongs to the family of mitochondrial solute carriers (MSCs) involved in the transport of a wide range of substrates across the inner mitochondrial membrane (Bashir *et al.*, 2011). Homologous mitochondrial iron importers have been identified in yeast (MRS3, MRS4) (Li and Kaplan, 2004), mouse (Paradkar *et al.*, 2009), *Drosophila* (Metzendorf and Lind, 2010), and zebrafish (mitoferrin) (Shaw *et al.*, 2006). The Arabidopsis chloroplast Fe-importing permease PIC1 is localized in the inner membrane and has cyanobacterial origin (Duy *et al.*, 2007).

In contrast to Fe importers, the proteins involved in the efflux of Fe from the mitochondria and plastids of plant cells have not yet been determined. Two mitochondrial proteins, Mmt1 and Mmt2, have been shown to be involved in the efflux of Fe from mitochondria in yeast (Li *et al.*, 2014). These proteins belong to the cation diffusion facilitator (CDF) family of divalent-metal transporters found in all kingdoms of life. A global phylogenetic analysis of CDF proteins from various organisms divided members of this family into three subgroups, namely Zn-CDF, Fe/Zn-CDF, and Mn-CDF, based on their putative specificity to the metal ions transported (Montanini *et al.*, 2007). Based on this analysis, the yeast Mmt1 and Mmt2 proteins fall into the Fe/Zn-CDF subgroup. The homologous protein has been found in plants and named MTP6, but its function in iron/zinc transport has not yet been confirmed.

In this study, we investigated the function of the MTP6 protein in cucumber. Using yeast and protoplasts isolated from Arabidopsis cells, we found that CsMTP6 localizes to mitochondria and contributes to the mitochondrial efflux of Fe and Mn. *CsMTP6* is ubiquitously expressed in cucumber organs, but the level of transcript and CsMTP6 protein is significantly increased in conditions of Fe deficiency or excess. These results indicate that plant MTP6 proteins contribute to the redistribution of Fe and Mn between the cytosol and mitochondria of plant cells, and undergo Fe-mediated transcriptional regulation to maintain mitochondrial and cytosolic iron homeostasis under varying conditions of Fe availability.

## Material and Methods

### Plant material and growth conditions

Seeds of cucumber (*Cucumis sativus* cv Krak) were germinated in darkness for 3 d on moist filter paper. The germinated seeds were transferred to hydroponic media containing a control nutrient solution (Migocka *et al.*, 2011) or solutions additionally supplemented with 10 μM MnCl_2_ or 1 mM FeSO_4_-EDTA, or solutions completely lacking in Mn or Fe. The Fe-free media were additionally supplemented with 100 μM of the Fe chelator bathophenanthroline disulfonate (BPS) to remove any contamination. Plants were grown for 2 weeks in a controlled environment with a day/night regime of 16/8 h (180 µmol m^–2^ s^–1^) and temperature of 24/22 °C. The media were continuously aerated and changed twice during the time of cultivation.

RETRACTED

### RNA extraction and real-time PCR

Total RNA was isolated from cucumber organs using TRI Reagent (Sigma), according to manufacturer’s instructions. RNA samples (2 µg) were reverse-transcribed using a High-Capacity cDNA synthesis kit (Applied Biosystems) and subjected to real-time PCR with primers specific for *CsMTP6* (forward primer 5′- TGGGATACAGATTCCACCGT -3′ and reverse primer 5′- TGCTCTTGGGATCATCATAAATTCCTA -3′) and for the reference gene encoding clathrin adaptor complex subunit CACS (forward primer 5′- GTGCTTTCTTTCTGGAATGC-3′ and reverse primer 5′- TGAACCTCGTCAAATTTACACA-3′). Amplification reactions were performed on a Lightcycler 480 (Roche) in a final reaction volume of 20 μl containing 2 μl of cDNA, 10 μl of 2× Real Time 2×PCR Mix SYBR (A&A Biotechnology), and 2 μl of each primer (10 µM) under the following conditions: 95 °C for 30 s, followed by 45 cycles of denaturation at 95 °C for 10 s, annealing at 60 °C for 10 s, and extension at 72 °C for 15 s. For the analysis of real-time PCR data, the relative gene expression was calculated using critical point (*C*p) values, which were converted into relative expression values according to the ΔΔ*C*_T_ method.

### Cloning of *CsMTP6*

The cDNA corresponding to *CsMTP6* was cloned by PCR amplification. Total RNA was isolated from the roots of 2-week-old cucumber seedlings that had been grown in standard liquid medium. cDNA was synthesized from the DNase-treated RNA using the SuperScript III (Invitrogen) and oligo-dT primers. For heterologous expression in yeast (*Saccharomyces cerevisiae*), the coding sequence of the *CsMTP6* gene (1500 bp without the stop codon) was amplified from cDNA as the *SpeI*-*SalI* fragment using the forward primer 5′-AAA*ACTAGT*ATGGGATACAGATTCCACCGTCT-3′ and the reverse primer 5′-TTT*GTCGAC*GTGGCTG AGCTGTGGAATTTGT-3′ (restriction sites in italics) and subcloned into the *SpeI* and *SalI* sites of the pUG35 vector (Niedenthal *et al.*, 1996) harboring the URA selective marker, a constitutive MET25 promoter, and the green fluorescent protein (GFP) reading frame located at the 3′-end of the multiple cloning site, to yield C-terminal GFP fusions. For the protein localization assay in protoplasts, the *CsMTP6* cDNA was amplified with the 5′-AAA*CTCGAG*ATGGGATACAGATTCCACCGT-3′ forward primer and the 5′-TTTA*CTAGTG*TGGCT GAGCTGTGGAATTT-3′ reverse primer to yield the *Xho*I-*SpeI* fragment, which was subcloned into pA7-GFP vector (Voelker *et al.*, 2006) to yield the C-terminal GFP fusion under the control of CaMV 35S promoter. The fidelity of all the constructs was established by sequencing.

RETRACTED

### Yeast strains, media, and fluorescence imaging

The yeast strains used in this study are listed in Table S1 at the Dryad Digital Repository (http://dx.doi.org/10.5061/dryad.306sf0b;Migocka *et al.*, 2018*b*). The strains were maintained in YPD liquid medium [2% (w/v) glucose, 2% (w/v) bactopeptone, and 1% (w/v) yeast extract]. All yeast transformations were performed as described previously (Migocka *et al.*, 2014), and the transformants were selected on complete synthetic media lacking uracil (SC–Ura), leucine (SC–Leu), or uracil and leucine (SC–Ura–Leu), containing 0.67% (w/v) yeast nitrogen base without amino acids (Difco), 2% (w/v) glucose, the required amino acids, and 2% (w/v) agar. The mitochondrial localization of CsMTP6 in yeast mitochondria was determined using a fluorescence microscope (Axio Imager M1, Carl Zeiss) equipped with a 100× oil-immersion objective. The cells were incubated with 100 nM MitoTracker Red (Molecular Probes) for 15 min prior to fixation to label the mitochondria.

### Immunolocalization of CsMTP6 in cucumber cells

Total microsomes were prepared from cucumber roots according to the procedure previously described by Kabała and Kłobus (2001). Tonoplast-enriched fractions were separated from the microsomal pellet in a discontinuous sucrose density gradient (the interphase between 20/28% sucrose) as described previously (Kabała and Kłobus, 2001). The right-side-out plasma membrane vesicles were separated from the microsomes in an aqueous dextran–polyethylene glycol two-phase system, following previously described methods (Larsson *et al.*, 1987; Migocka *et al.*, 2011). Crude mitochondria- and plastid-enriched fractions were prepared from cucumber roots essentially as described by Vigani *et al.* (2013). Purified mitochondrial fractions were collected from the 28/40% interface of a Percoll gradient following centrifugation of crude mitochondrial pellets on a 40, 28, and 13.5% (v/v) Percoll step-gradient (Vigani *et al.*, 2013). The distribution of marker membrane proteins in each membrane fraction was examined by western blot analysis with specific antibodies (Agrisera, Vännäs, Sweden) raised against the plasma membrane (PM) H^+^-ATPase (AS07 260), the tonoplast V-ATPase (epsilon subunit) (AS07 213), the mitochondrial COXII cytochrome oxidase (AS04 053A), and the plastidial outer-envelope membrane translocon complex Toc75 (AS06 150). Immunolocalization of CsMTP6 was carried out using a specific antibody raised against a synthetic peptide antigen corresponding to the predicted C-terminal sequence of CsMTP6 (positions 324–337, C+CEGVKGCHRLRGRRA; C, additional cysteine residue for linkage with keyhole limpet hemocyanin KLH). The peptide conjugated to KLH was injected into two rabbits (three immunizations per rabbit). The CsMTP6-specific IgG was purified using Sepharose resin linked with the antigen peptide, and the purified antibody was detected and quantified by an ELISA test. The peptide antigen and the antibody were synthesized by GeneScript (Piscataway, NJ, USA). Western blot analysis was performed essentially as described previously by Migocka *et al.* (2011) with a 1:1000 dilution of primary antibodies for CsMTP6, a 1:5000 dilution of the primary antibodies for marker membrane proteins, and a 1:20 000 dilution of the secondary anti-rabbit IgG antibody conjugated to horseradish peroxidase (AS09 602, Agrisera). The blots were developed using an enhanced chemiluminescence system (ChemiDocTMMP Imaging System, Bio-Rad).

RETRACTED

### Metal and H_2_O_2_ sensitivity spot assays

For metal and H_2_O_2_ tolerance assays, serial dilutions (OD_600_ 0.1, 0.01, and 0.001) of cells grown overnight were spotted onto agar plates containing selective media supplemented with different concentrations of heavy metals (FeSO_4_-EDTA, CoCl_2_, CuSO_4_, MnCl_2_, CdCl_2_), H_2_O_2_, or 100 μM iron chelator BPS (low-Fe media). Plates were incubated at 30 °C for 3–4 d prior to imaging.

### Cytosolic gentisate 1,2-dioxygenase assays

The cytosolic gentisate 1,2-dioxygenase (*c-GDO*)*-FLAG* fragment was amplified from the pRS426 vector using the forward primer 5′- ATTAACAAG *GCCATTACGGC C*AAAAA TGCAGAACG AAAAACT CGACCAC-3′ and the reverse primer 5′- AACTGATT *GGCCGAGGCGGCC* TCACTTGTCGTCATC GTCTTTGTAGTC-3′ introducing two *SfiI* sites (in italics), respectively, and subcloned into the *SfiI*-*SfiI* sites of the yeast expression vector pBT3C carrying a *Leu* selectable marker (Dualsystems Biotech). The pBT3C-GDO plasmid was then transformed into yeast cells harbouring plasmids pUG35 or pUG35-CsMTP6, and the transformants carrying two vectors were selected on SC–Ura–Leu solid media. Cells were grown overnight to mid-log phase in liquid SC–Ura–Leu medium and then for 8 h in the same fresh medium supplemented with 100 μM FeSO_4_-EDTA. Following this treatment, cells were homogenized using glass beads in 25 mM Tris-HCl, pH 7.4, 50 mM NaCl, and 0.5 mM phenylmethanesulfonyl fluoride (Sigma-Aldrich). The presence of c-GDO in the extract was confirmed by western blot analysis using antibodies against FLAG (1:10 000, Sigma Aldrich). c-GDO activity was measured spectrophotometrically at 340 nm as described previously (Li *et al.* 2014), in an assay mixture containing 20 mM Tris-HCl (pH 8.0) and 0.1 mM 2,3-dihydroxy-benzoic acid (gentisic acid) (Sigma-Aldrich). Enzyme activity was calculated using an extinction coefficient of 10.2 cm^−1^mm^−1^ and was expressed as nmol of substrate converted per minute per mg of protein.

RETRACTED

### Mn-SOD assays

For determination of Mn-SOD activity, mitochondria prepared from yeast cells or protoplasts were disrupted by freeze–thaw cycles and suspended in 20 mM HEPES, 1 mM EDTA, 250 mM sucrose, and 0.1% Triton X-100 to release enzymes (Lanza and Nair, 2009). Mn-SOD activity was measured by activity assays essentially as described previously by Weydert and Cullen (2010), using xanthine-xanthine oxidase to generate O_2_^•−^ and nitroblue tetrazolium (NBT) reduction as an indicator of O_2_^•−^ production. This assay allows for the indirect determination of Mn-SOD activity based on competition between SOD and NBT, which is reduced by superoxide into blue formazan and results in a measurable change in absorption. The reaction was measured spectrophotometrically at 560 nm using a UV/VIS Carry 100 spectrophotometer (Agilent Technologies). As CuZn-SOD has also been shown to be present in the intermembrane space of mitochondria (Okado-Matsumoto and Fridovich, 2001; Sturtz *et al.*, 2001), an inhibitor, 5 mM potassium cyanide, was added to the reaction assays to completely inactivate CuZn-SOD activity (Asada *et al.*, 1974). One unit of Mn-SOD activity was defined as the amount of enzyme required for the inhibition of the NBT reduction rate to half of the maximum. The specific activity of Mn-SOD was expressed in units per mg protein.

### Transformation of Arabidopsis protoplasts and confocal imaging

Arabidopsis cell suspension protoplasts were isolated and transformed essentially as described previously (Thomine *et al.*, 2003). Following transformation, the protoplasts were incubated in the dark at 23 °C for 2–3 d. Confocal fluorescence images were acquired 24–36 h after transformation using an Olympus FluoView FV1000 (lens, Olympus UPlanSApo 60×/1.35 oil; filter, BF490-590) with excitation at 473 nm. Mitochondria of the protoplasts were counterstained with 25 nM MitoTracker Red CMXRos (Molecular Probes) for 15–60 min.

### Mitochondria preparation from Arabidopsis protoplasts

Mitochondria were prepared from Arabidopsis cell suspension protoplasts essentially as described previously by Nishimura *et al.* (1982), with slight modifications. To measure the accumulation of Fe or Mn in the mitochondria, the transformed protoplasts (2 ml) were incubated with 100 μM FeSO_4_-EDTA or 100 μM MnSO_4_ for 12 h in darkness with a slow flotation prior to preparation. The metal-treated protoplasts were gently washed twice with a 10 mM MOPS-KOH buffer (pH 7.2), containing 0.34 M glucose, 0.34 M mannitol, and 1 mM EDTA, and finally suspended in 30 ml of homogenization buffer, consisting of 10 mM MOPS-KOH buffer (pH 7.2), 0.3 M mannitol, 1 mM EDTA, 0.1% defatted BSA, and 0.6% PVPP. Homogenization was achieved by a mechanical disruption of protoplasts in a glass homogenizer (3-cm diameter) with 10 gentle strokes, and the resulting homogenate was centrifuged at 1000 *g* for 10 min to pellet the plastids and aggregated organelles. The supernatant was centrifuged at 10 000 *g* for 10 min and the pellet obtained was gently suspended in 1 ml of a buffer containing 10 mM MOPS-KOH buffer (pH 7.2), 0.3 M mannitol, and 1 mM EDTA. The suspension was layered on top of a discontinuous Percoll density gradient composed of 60/45/28/5% (v/v) Percoll in 20 mM MOPS-KOH buffer (pH 7.2), 0.25 M sucrose, and 1 mM EDTA, and centrifuged for 30 min at 30 000 *g*. Following centrifugation, the plastidial (28/5% interphase) and mitochondrial (45/28% interphase) fractions were collected and subjected to western blot analysis with antibodies raised against Toc75, COXII, and GFP to confirm the purity of the mitochondrial fraction and the presence of CsMTP6 in mitochondrial membranes.

RETRACTED

### Mitochondria preparation from yeast cells

To determine the metal content in yeast mitochondria, cells transformed with the pUG35 plasmid carrying *CsMTP6* or with the empty vector were grown for 48 h in a SC/Glu–Ura medium and then for 12 h in the same media supplemented with 100 µM of the selected metals (FeSO_4_-EDTA, CdCl_2_, NiCl_2_, MnSO_4_, CoCl_2_, CuCl_2_, ZnSO_4_). Highly purified mitochondria were isolated from yeast cells as described previously (Gregg *et al.*, 2009) using a four-step sucrose gradient (60/32/23/15%). The intact mitochondria were collected from the 60/32% sucrose interface and subjected to western blot analysis with anti-CsMTP6 antibodies to confirm the presence of CsMTP6 in mitochondrial membranes.

### Determination of mitochondrial heavy metal content

Mitochondria prepared from protoplasts or yeast cells were digested with concentrated HNO_3_ at 160 °C for 2 h. The heavy metal content (Fe, Mn, Cu, Zn, Ni, Co, Cd) was measured by flame atomic absorption spectrometry (AAS).

### Protein determination

Protein contents of all the membrane fractions were determined using Bradford assays (Bradford, 1976).

RETRACTED

### Bioinformatics and accession number

The predicted full coding sequence of *CsMTP6* was retrieved from GenBank as described previously (Migocka *et al.*, 2014). The putative CsMTP6 transmembrane domains were predicted using HMMTOP (Tusnády and Simon, 2001) and visualized in TMRPres2.D (Spyropoulos *et al.*, 2004). The mitochondrial targeting peptide was identified using MitoProt II, v1.101 (https://bio.tools/MITOPROT_II, last accessed on October 19, 2018). The nucleotide and the putative amino acid sequences of CsMTP6 are available in GenBank under the accession number KX118275.

### Statistical analysis

Student’s *t*-tests, Tukey’s test, and ANOVA (MS Excel) were used for statistical analyses.

## Results and discussion

### Sequence and expression analysis of CsMTP6

The plant MTP family has been divided into seven groups (1, 5, 6, 7, 8, 9, and 12) based on annotated MTP sequences from Arabidopsis (Gustin *et al.*, 2011). These groups form the three primary clades of the CDF family that differ in their putative substrate specificity: Zn-CDF, Fe/Zn-CDF, and Mn-CDF. Group 6 containing the MTP6 proteins has been classified in the Fe/Zn-CDF group, including bacterial FieF-like and WmFieF-like proteins and the fungal MMT-like proteins, which are involved in Fe transport (Li and Kaplan, 1997; Grünberg *et al.*, 2001; Grass *et al.*, 2005; Li *et al.*, 2014). The genes encoding plant MTP6 proteins have been identified in all the plant genomes sequenced so far except for the those of the red alga *Cyanidioschyzon merolae*, and the green algae *Ostreococcus tauri*, *O. lucimarinus*, and *Chlamydomonas reinhardtii*, suggesting that the members of group 6 in algae have been lost (Gustin *et al.*, 2011). A gene encoding a protein bearing a close similarity to MTP6-like protein has also been identified in the genomes of the cucumber cultivars Chinese long (acc. no. ACHR01000689) and Borszczagowski (acc. no. ACYN01005409) (Migocka *et al.*, 2014). FGENESH (Find GENES HMM), a Hidden Markov Models (HMM)-based *ab initio* gene-structure prediction program (Salamov and Solovyev, 2000) was used to identify the transcription site, exon/intron boundaries, and the polyadenylation signal sequence of the *CsMTP6* gene in these two cultivars and it determined that the cucumber *CsMTP6* gene contains 13 exons and 12 introns and encodes a putative protein of 528 amino acids (Migocka *et al.*, 2014). Based on the sequence retrieved from GenBank, we designed two specific primers to analyse *CsMTP6* expression in the different organs of the cucumber cultivar Krak. *CsMTP6* was differentially expressed in all the vegetative organs, with the lowest expression level in the hypocotyls (Fig. S1, Dataset S1 at Dryad). cDNA prepared from the bulk sample of roots was used to amplify the full cDNAs of *CsMTP6* for the subsequent analysis of CsMTP6 function and localization in yeast and Arabidopsis protoplasts. Comparative analysis of the cDNA generated *in silico* and the cDNA amplified by PCR revealed the lack of 84 nucleotides encoding a 24-amino acid fragment NLAIILSESQCFQGSRNLAWPSLFSCKQ in the amplified *CsMTP6* product (Fig. S2A, B at Dryad). There are three possible reasons for this discrepancy: first, the prediction of the *CsMTP6* cDNA by FGENESH might be inaccurate; second, the difference in *CsMTP6* cDNA and protein sequences between the cucumbers Chinese long, Borszczagowski, and Krak may result from a mutational event and reflect some genetic variability between different cultivars; or third, alternative splicing of *CsMTP6* mRNA might occur, giving rise to more than one transcript. Splicing variants of *AtMTP3*, *AtMTP5*, *AtMTP6*, and *AtMTP9* have already been reported and submitted to the Arabidopsis Information Resource (TAIR) database (https://www.arabidopsis.org, last accessed on October 19, 2018) and the plant membrane protein database Aramemnon (http://aramemnon.uni-koeln.de/index.ep, last accessed on October 19, 2018). In addition, the existence of multiple transcripts of the *MTP1* gene has been reported in the heavy metal hyperaccumulator *Thlaspi goesingense* (*TgMTP1t1* and *TgMTP1t2*) (Persans *et al.*, 2001). In order to confirm the structure of the *CsMTP6* transcript and identify its possible alternative splicing variants, we analysed the reassembled genome of the cultivar Chinese long (available at http://cmb.bnu.edu.cn/Cucumis_sativus_v20/, last accessed on October 19, 2018), which was reannotated with RNA-Seq reads from poly(A) RNAs obtained from 10 cucumber tissues (Li *et al.*, 2011). We searched the database for the *CsMTP6* gene and found only one transcript annotated as *Csa7G395210.1*, consisting of 12 exons. The alignment of this transcript and the PCR-amplified *CsMTP6* cDNA of the Krak cultivar showed the same length (1503 bp) and 100% identity of both protein-coding sequences (Fig. S2C at Dryad). These results indicated that only one *CsMTP6* transcript was present in the cucumber tissues examined and suggested that the differences in the transcripts amplified by PCR and predicted *ab initio* (Fig. S2A at Dryad) resulted from the inaccuracy of the FGENESH prediction.

RETRACTED

*In silico* analysis of the amino acid sequence deduced from the PCR-amplified *CsMTP6* cDNA revealed the presence of four putative transmembrane helices (TMs) and the mitochondrial targeting sequence (MTS) in the N-terminal domain of CsMTP6 (Fig. 1). The signature sequence characteristic for CDF proteins covered the amino acids 104– 147 located within the first TMI helix and the loop connecting helices TMI and TMII of CsMTP6 (Fig. 1). The two Fe/Zn group-specific motifs were identified in the putative TMI helix (*H*SVS*D*) and in the loop connecting helices TMIII and TMIV (*H*HRA*D*) (Fig. 1). Based on the X-ray structure of the *E. coli* YiiP (EcFieF) (Lu and Fu, 2007), the conservative amino acids from both motifs (HD-HD in CsMTP6) are thought to form metal-binding sites. Interestingly, both motifs are located in the transmembrane helices II and V of YiiP (Lu and Fu, 2007). The predicted topology of CsMTP6 (4 TMHs) was quite different from the topology of typical CDF transporter (6 TMHs) (Montanini *et al.*, 2007) and this difference could be a reason for the presence of the HHRAD motif out of the CsMTP6 TMH. However, this predicted topology needs to be experimentally verified to confirm the presence of both motifs in or out of the transmembrane helices. In addition, we did not identify a His-rich region typical for the members of CDF family in CsMTP6 (Montanini *et al.*, 2007). Instead, CsMTP6 had a histidine/serine-rich loop located between TMHs II and III that is typical for sequences belonging to Zrg17-like and MMT-like clusters (Montanini *et al.*, 2007) (Fig. 1).

**Fig. 1.** Sequence analysis of cucumber CsMTP6. The transmembrane topology of CsMTP6 was predicted by HMMTOP. The positions of CDF signature sequence, mitochondrial targeting peptide, and HD motif 2 are indicated by dashed arrows. The two motifs specific for the Fe/Zn-subgroup, HSVSD (motif HD 1 in the CDF signature sequence) and HHRAD (motif HD 2) are highlighted in boxes. The amino acids of the HD motifs are marked in bold and the conservative histidine and aspartate are underlined.

### CsMTP6 localizes to the mitochondria

To confirm the mitochondrial localization of CsMTP6, we tagged the green fluorescent protein (GFP) to the C-terminus of CsMTP6 and investigated the subcellular localization of this fusion protein in protoplasts isolated from Arabidopsis suspension cells. Protoplasts transformed with the *CsMTP6-GFP* fusion were stained with MitoTracker-Red to simultaneously visualize the mitochondria. As shown in Fig. 2A, the protoplasts containing CsMTP6-GFP displayed dotted green fluorescence signals, which clearly overlapped the regions stained with MitoTracker, confirming that CsMTP6 localizes to the mitochondria. To further confirm this localization in cucumber cells, we performed immunolocalization of CsMTP6 in different subcellular fractions prepared from roots using a specific anti-CsMTP6 antibody. Western blot analysis of the fractions enriched in plasma membranes, tonoplasts, plastids, or mitochondria revealed a specific band migrating at a molecular mass of 35 kDa only in the mitochondrial fractions, consistent with the results obtained from protoplast imaging (Fig. 2B). In comparison, no immunoreactive bands were detected for the other membrane fractions of the cucumber cells. The observed molecular mass was lower than that predicted from the deduced amino acid sequence (~50 kDa), suggesting that the target peptide is removed following the targeting of CsMTP6 to the mitochondrial membrane. To date, members of the plant MTP family have been found to be localized to the tonoplast (Delhaize *et al.*, 2003; Kobae *et al.*, 2004; Arrivault *et al.*, 2006; Migocka *et al.*, 2014, 2015*a*), the Golgi/prevacuolar system (Delhaize *et al.*, 2007; Peiter *et al.*, 2007; Pedas *et al.*, 2014; Fujiwara *et al.*, 2015), or the plasma membrane (Migocka *et al.*, 2015*b*; Ueno *et al.*, 2015). The only members of the CDF family that have been found localized to the mitochondria include the two CsMTP6 homologs from yeast, ScMMT1 and ScMMT2 (Li and Kaplan, 1997; Li *et al.*, 2014), suggesting that the yeast and plant members of the Fe/Zn-CDF group can fulfill similar physiological functions. It has been shown that the yeast ScMMT1 and ScMMT2 proteins contribute to the export of Fe from the mitochondria (Li *et al.*, 2014). In order to determine the metal specificity of CsMTP6, we examined the effects of *CsMTP6* expression in yeast deficient in different heavy metal transporters.

RETRACTED

**Fig. 2.** Subcellular localization of CsMTP6. (A) Mitochondrial localization of CsMTP6 in protoplasts prepared from suspensions of *Arabidopsis* cells: 1, GFP fluorescence of protoplast expressing CsMTP6-GFP; 2, MitoTracker red fluorescence; 3, merged image; 4, transmission image of the same protoplast. The scale bar is 10 µm. (B) Immunolocalization of CsMTP6 in cucumber root cells. SDS-PAGE followed by western blot analysis of plasma membrane (PM), tonoplast (Ton), and mitochondrial (Mit) and plastidial (Plast) fractions. The fractions (15 μg of protein per lane) were blotted with the primary antibodies to identify marker enzymes for the plasma membrane (PM-ATPase), tonoplast (V-ATPase), plastids (Toc75), mitochondria (COXII), and to localize CsMTP6. L, protein ladder.

### *CsMTP6* expression affects Fe homeostasis in yeast with deletion of mitochondrial iron transporters

Since all the members of Fe/Zn-CDF characterized to date contribute to Fe transport, we first investigated whether CsMTP6 is involved in the transport of Fe when expressed in yeast cells. over the last few years, a range of organelle Fe transporters have been identified in yeast cells that contribute to cellular homeostasis. These include the MRS3 and MRS4 proteins involved in the mitochondrial Fe import (Mühlenhoff *et al.*, 2003), the vacuolar Fe transporter CCC1 (Li *et al.*, 2001), and the MMT1 and MMT2 proteins involved in mitochondrial Fe export (Li *et al.*, 2014).

RETRACTED

The MRS3/4 proteins are members of the mitochondrial solute carrier family that catalyse the transport of Fe into the mitochondria along a concentration gradient (Froschauer *et al.*, 2009; Mühlenhoff *et al.*, 2003), whereas CCC1 is a member of the vacuolar iron transporters (VIT) family involved in the transport of Fe^2+^ and Mn^2+^ into the vacuole, probably by a H^+^ antiport carrier-type mechanism (Li *et al.*, 2001; Kim *et al.*, 2006). In yeast, the CCC1-mediated transport of Fe into the vacuole is the main mechanism of Fe detoxification and tolerance (Li *et al.*, 2001). Deletion of genes encoding MRS3/4 and CCC1 results in two different iron-dependent phenotypes, exhibiting increased sensitivity to low Fe (*Δmrs3Δmrs4*) due to the impaired import of Fe into the mitochondria, or increased sensitivity to high Fe (*Δccc1*), resulting from the impaired export of Fe from the cytosol into the vacuole (Li *et al.*, 2001, 2014; Mühlenhoff *et al.*, 2003). The expression of *CsMTP6* in both yeast mutants did not complement their Fe-dependent phenotypes (Fig. 3A). Furthermore, the CsMTP6-GFP fusions were observed to co-localize with the mitochondrial networks of both *Δccc1* and *Δmrs3Δmrs4* cells (Fig. 3B). Mitochondrial localization and the lack of complementation of the *Δccc1* and *Δmrs3Δmrs4* mutations by CsMTP6 indicated that the cucumber protein was not involved in the sequestration of Fe into the vacuole under high Fe conditions or in the import of Fe into the mitochondria under low Fe conditions.

**Fig. 3.** Complementation assay and localization of CsMTP6 in yeast cells defective in vacuolar and mitochondrial iron transporters. (A) Representative images (from four replicates) of serial dilutions of the wild-type (WT) and yeast mutants sensitive to high iron (*Δccc1*) or low iron (*Δmrs3mrs4* and *Δmmt1/mmt2*) transformed with the empty vector or with *CsMTP6*. Yeast were grown in SC/Glu–Ura media supplemented with 100 µM BPS (low Fe), 3 mM FeSO_4_-EDTA, or in the control SC/Glu–Ura media. (B) CsMTP6-GFP localization in *Δccc1*, *Δmrs3mrs4* and *Δmmt1/mmt2* cells. Yeast cultured overnight in control liquid SC/Glu–Ura media were diluted to OD_600_ 0.1 and then grown in liquid SC/Glu–Ura media supplemented with 3 mM FeSO_4_-EDTA (*Δccc1*) or 100 µM BPS (low Fe, *Δmrs3mrs4* and *Δmmt1/mmt2*) for 8–10 h. 1, Transmission image of the cells expressing CsMTP6-GFP; 2, GFP fluorescence; 3, MitoTracker red fluorescence; 4, merged image. Scale bars are 5 μm.

RETRACTED

Since plant MTP6-like proteins belong to the same phylogenetic cluster as the yeast mitochondrial MMT1 and MMT2 proteins, we expected that the expression of *CsMTP6* would complement the *Δmmt1Δmmt2* mutation or result in the same phenotypes observed when MMT1 and MMT2 are overexpressed. It has been shown previously that a deletion of MMT1 and MMT2 in yeast has no effect on Fe toxicity but results in a decrease in cytosolic Fe and an increased sensitivity to Fe deficiency (Li *et al.*, 2014). The decreased growth of the yeast strain *Δmmt1Δmmt2* in Fe-free media is thought to result from the inability of this mutant to use mitochondrial Fe (i.e. to export Fe from mitochondria) under starvation conditions (Li and Kaplan, 1997). As shown in Fig. 3A, the expression of *CsMTP6* in *Δmmt1Δmmt2* cells reversed the effect of the mutation and rendered the double-mutant more resistant to Fe deficiency. Similar to the *Δccc1* and *Δmrs3Δmrs4* strains, the CsMTP6-GFP fusion co-localized with the mitochondrial network of the yeast *Δmmt1Δmmt2* mutant (Fig. 3B), confirming that CsMTP6 could restore the mitochondrial Fe export in *Δmmt1Δmmt2* cells.

To further support the hypothesis that CsMTP6 contributes to the transport of Fe out of the mitochondria, we examined the effects of *CsMTP6* expression on the mitochondrial and cytosolic Fe content in wild-type yeast and in the cells deleted for MMT1 and MMT2. Cytosolic Fe was determined based on the activity of cytosolic gentisate 1,2-dioxygenase (c-GDO) following the transformation of cells expressing *CsMTP6* with a *c-GDO*-expressing plasmid. c-GDO is absent in yeast; however, when expressed in yeast, it localizes only in the cytosol and shows Fe^2+^-dependent activity using gentisate as a substrate, and therefore the activity of this enzyme can be used as a measure of cytosolic Fe (Li *et al.*, 2014). The presence of CsMTP6 and c-GDO in yeast was confirmed by western blot analysis (Fig. 4A). Mitochondria isolated from yeast transformants showed major immunoreactive bands migrating just below 70 kDa (Fig. S3 at Dryad), corresponding to the CsMTP6-GFP fusion proteins (~35 kDa for CsMTP6 + 27 kDa for GFP). As shown in Fig. 4B and Dataset S2 at Dryad, the deletion of MMT1 and MMT2 in yeast resulted in a decrease in cytosolic Fe, observed as a decrease in c-GDO activity. In contrast, the mitochondrial Fe content of *Δmmt1Δmmt2* cells was increased (Fig. 4C, Dataset S3 at Dryad), confirming the function of MMT proteins in mitochondrial Fe export. Expression of *CsMTP6* in wild-type yeast cells markedly increased c-GDO activity and significantly decreased mitochondrial Fe content (Fig. 4B, C, Datasets S2, S3 at Dryad), indicating that CsMTP6 supported endogenous MMT1 and MMT2 proteins in the transport of Fe from the mitochondria to the cytosol. Consistent with this hypothesis, the expression of *CsMTP6* in the *Δmmt1Δmmt2* mutant reversed the effect of the mutation and restored the mitochondrial and cytosolic Fe levels to those observed in wild-type cells (Fig. 4B, C, Datasets S2 and S3 at Dryad), confirming that the cucumber protein complements the lack of MMT1 and MMT2 and contributes to the transport of Fe out of the mitochondria.

RETRACTED

**Fig. 4.** Cytosolic and mitochondrial Fe content in yeast expressing *CsMTP6*. (A) Western blot analysis of CsMTP6-GFP and c-GDO with a carboxyl-FLAG epitope in wild-type (WT) yeast and transformants using antibodies against GFP and FLAG; vec, empty vector. (B) c-GDO activity in WT and yeast mutant cells expressing CsMTP6-GFP and GDO-FLAG. c-GDO activity is expressed as nmol of substrate converted min^–1^ mg^–1^ of protein. Data are means (±SD) of four individual transformants. (C) Mitochondrial Fe content in yeast expressing *CsMTP6*. Data are means (±SD) of three separate experiments. Significant differences were determined using Tukey’s test.

### *CsMTP6* expression affects the sensitivity of yeast to copper, cobalt, and H_2_O_2_

To further confirm that CsMTP6 can be a functional homolog of the yeast proteins MMT1 and MMT2, we investigated the effect of *CsMTP6* expression on yeast sensitivity to copper, cobalt, and H_2_O_2_. Previous studies have shown that overexpression of *MMT1* and *MMT2* in wild-type yeast decreases cobalt sensitivity and increases copper and H_2_O_2_ sensitivity (Li *et al.*, 2014). In contrast, cells deleted for *MMT1* and *MMT2* are significantly more sensitive to Co, and moderately more resistant to Cu (Li *et al.*, 2014). The expression of *CsMTP6* in wild-type yeast resulted in a cobalt-resistant phenotype (Fig. 5A) similar to that observed in yeast overexpressing *MMT1* and *MMT2* (Li *et al.*, 2014). In addition, the expression of *CsMTP6* in *Δmmt1Δmmt2* cells suppressed their Co-sensitive phenotype (Fig. 5A). The response of the yeast mutant to cobalt stress could have resulted from the CsMTP6-induced modification of the cytosol Fe level. It has been well documented in yeast that cobalt stress immediately and dramatically induces the expression of genes involved in Fe uptake (Stadler and Schweyen, 2002). This response is mediated by the Aft1 transcriptional factor, which accumulates in the nucleus under Fe starvation and Co excess and activates a set of genes involved in Fe uptake and homeostasis (termed the iron regulon) (Stadler and Schweyen, 2002). Consequently, yeast cells deleted for *AFT1* are more sensitive to Co, and this Co-sensitive phenotype is not complemented by the overexpression of *MMT1* and *MMT2*, indicating that AFT1 and not MMT1 and MMT2 is required for Co resistance (Li *et al.*, 2014). The expression of *CsMTP6* in *Δaft1* cells also did not complement the Co-sensitive phenotype of this mutant strain (Fig. 5A), suggesting that CsMTP6 may not be directly involved in Co transport in yeast cells. Consistent with this hypothesis, the mitochondrial Co content in yeast expressing *CsMTP6* was not affected by the activity of the cucumber protein (Fig. 5B, Dataset S3 at Dryad). However, since we did not perform direct measurements of heavy metal transport, additional studies are required to verify the ability of CsMTP6 to transport Co.

RETRACTED

**Fig. 5.** Effect of *CsMTP6* expression on yeast sensitivity to Co, Cu, and H_2_O_2_. (A) Representative images (from four replicates) of serial dilutions of the wild-type (WT) and *Δmmt1Δmmt2* and *Δaft1* mutants transformed with the empty vector or *CsMTP6* and grown on either SC/Glu–Ura medium supplemented with 2 mM CoCl_2_ or control SC/Glu–Ura medium. (B) Mitochondrial Co content in yeast expressing *CsMTP6*. Data are means (±SD) from three separate experiments. (C) Representative images (from four replicates) of serial dilutions of the WT and *Δmmt1Δmmt2* mutants transformed with the empty vector or *CsMTP6* and grown on either SC/Glu–Ura medium supplemented with 1.5 mM CuCl_2_ or control SC/Glu–Ura medium. (D) Representative images (from four replicates) of serial dilutions of the WT and *Δfet5Δsmf3* mutants transformed with the empty vector or *CsMTP6* and grown on either SC/Glu–Ura medium supplemented with 0.0075% H_2_O_2_ or control SC/Glu–Ura medium. (E) Mitochondrial Cu content in yeast expressing *CsMTP6*. Data are means Cu l(±SD) from three separate experiments.

Similar to *MMT1* and *MMT2* overexpression, the expression of *CsMTP6* in yeast resulted in Cu-sensitive and H_2_O_2_-sensitive phenotypes of the wild-type, a Cu-sensitive phenotype of the *Δmmt1Δmmt2* mutant, and a H_2_O_2_-sensitive phenotype of the *Δfet5Δsmf3* mutant, resulting from a deletion of vacuolar the Fe exporters FET5/SMF3 (Fig. 5C, D). Similar to Co, the mitochondrial Cu content in yeast was not affected by CsMTP6 activity (Fig. 5E, Dataset S3 at Dryad). As has already been shown in yeast, increased cytosolic Fe resulting from the overexpression of *MMT1* and *MMT2* significantly raises the level of cellular oxidants and leads to increased oxidant damage in cells (Li *et al.*, 2014). These results suggest that the Cu- and H_2_O_2_-sensitive phenotypes of yeast expressing *CsMTP6* were caused by the changes in cellular redox homeostasis resulting from the CsMTP6-mediated increase in cytosolic Fe, and not by the contribution of the protein in Cu transport. Although the ability of CsMTP6 to transport Cu needs to be verified in direct transport assays, the similar phenotypes resulting from *MMT1* and *MMT2* overexpression or *CsMTP6* expression in yeast support the hypothesis that the plant and yeast homologs affect redox homeostasis in yeast in the same way.

RETRACTED

### *CsMTP6* expression affects the Mn-sensitive phenotype and the mitochondrial Mn level of the yeast mutant K667

A few characterized members of the Fe/Zn-CDF subgroup from bacteria, including FieF from *E. coli* (Grass *et al.*, 2005), MgMamB from *Magnetospirillum gryphiswaldense* (Grünberg *et al.*, 2001), and WmFieF from *Cupriavidus metallidurans* (Munkelt *et al.*, 2004), have been shown to be involved in the transport of other metals in addition to Fe, such as Zn^2+^, Co^2+^, Cd^2+^, and Ni^2+^. In order to determine the substrate specificity of CsMTP6, we further investigated whether it was able to complement the mutant phenotype displayed by yeast strains sensitive to Zn (*Δzrc1*), Cd, Mn, and Ni (K667, *Δpmc1Δvcx1Δcnb*), or Mn deficiency (Δ*smf1*). The presence of CsMTP6 in the mitochondria of all transformants was confirmed under fluorescence microscopy (Fig. S4 at Dryad). CsMTP6 did not affect the sensitivity of the *Δzrc1* and K667 cells to Zn, Ni, and Cd, and the mitochondrial contents of these metals were not affected by *CsMTP6* expression (Fig. S5, Dataset S3 at Dryad). These results suggest that CsMTP6 may not be capable of Zn, Ni, or Cd transport in yeast cells. In contrast, the expression of *CsMTP6* in the K667 strain fully complemented the Mn-sensitive phenotype and significantly reduced the mitochondrial Mn content and Mn-SOD activity of this yeast mutant (Fig. 6A–C, Dataset S3 at Dryad), suggesting that CsMTP6 may be involved in the transport of both Fe and Mn out of the mitochondria. Interestingly, the levels of metals determined in the mitochondria of yeast were quite high (nmol concentrations), indicating that they were able to tolerate a certain amount of Zn, Mn, Ni, or Cd. Taking into the consideration the metabolic processes occurring in mitochondria, it is assumed that organic acids (citrate, isocitrate, malate, aconitate, oxaloactetate) may be involved in the alleviation of heavy metal toxicity within them by forming Zn-citrate, Zn-malate, Ni-citrate, Cu-citrate, Mn-citrate, and Cd-citrate (Mathys, 1977; Glusker, 1980; Thurman and Rankin, 1982; Godbold *et al.*, 1984; Harrington *et al.*, 1996; Parker *et al.*, 2001). However, based on the results of our metal spot-test assays we may conclude that the capabilities of mitochondria to chelate Zn, Mn, Ni, or Cd are very limited.

RETRACTED

**Fig. 6.** Effect of *CsMTP6* expression on the Mn sensitivity, mitochondrial Mn content, and Mn-SOD activity of yeast. (A) Representative images (from four replicates) of serial dilutions of the wild-type (WT) and K667 mutants transformed with the empty vector or *CsMTP6* and grown on either SC/Glu–Ura medium supplemented with MnSO_4_ or control SC/Glu–Ura medium. (B) Mitochondrial content of Mn in yeast expressing *CsMTP6*. Data are means (±SD) from separate experiments. (C) Mitochondrial Mn-SOD activity in yeast expressing *CsMTP6*. Data are means (±SD) from three separate experiments, expressed as enzyme units (U). Significant differences were determined using Tukey’s test. (D) Representative images (from four replicates) of serial dilutions of the WT and Δ*smf1* mutants transformed with the empty vector or *CsMTP6* and grown on either SC/Glu–Ura medium supplemented with EGTA (low Mn medium) or control SC/Glu–Ura medium.

Although CsMTP6 complemented the high Mn-sensitive phenotype of the K667 strain, it did not restore the growth of Δ*smf1* cells in low-Mn media (Fig. 6D). Smf1p is a cell-surface transporter involved in high-affinity Mn uptake and trafficking in yeast cells, and therefore deletion of *SMF1* results in a decrease in the intracellular Mn concentration and increased sensitivity to the Mn chelator EGTA (Supek *et al.*, 1996). The inability of CsMTP6 to complement the sensitivity of Δ*smf1* to low Mn indicates that mitochondrial efflux is not able to complement the deficiency in Mn uptake of the mutant cells, or to induce transcriptional pathways that could increase the level of cellular Mn through enhanced influx across the plasma membrane or enhanced efflux from the vacuole. These results are consistent with previous data that indicate that the Mn regulatory pathways identified to date do not all occur at the transcriptional level, but instead also involve post-translational modifications of the localization and turnover or the Smf1p and Smf2p Mn transporters (Liu and Culotta, 1999; Portnoy *et al.*, 2000; Reddi *et al.*, 2009). As CsMTP6 localized in the mitochondria under Mn deficiency (Fig. S4 at Dryad), it was not able to catalyse uptake by Δ*smf1* cells. Furthermore, the concentration of Mn detected in the mitochondria of yeast cells was significantly lower compared to that of Fe (Figs 4C, 6B), indicating that their capacity to accumulate and tolerate Mn excess was more limited. Indeed, the complementation of the Mn-sensitive phenotype of K667 cells by CsMTP6 suggests that excess Mn negatively affects the mitochondria of yeast cells. The K667 mutant is deficient in the functional Ca^2+^‐dependent protein phosphatase calcineurin, the vacuolar Ca^2+^(Mn^2+^)/H^+^ exchanger Vcx1p (Mnr1), and the vacuolar Ca^2+^‐ATPase Pmc1p (Cunningham and Fink, 1996). Calcineurin is required for the activation of Mn^2+^/H^+^ transport activity by Vcx1p (Mnr1) and for the activation of the high‐affinity Ca^2+^/Mn^2+^‐transporting ATPase Pmr1p, and may also prevent the entry of excess Mn^2+^ into the cell (Farcasanu *et al.*, 1995; Lapinskas *et al.*, 1995; Pittman *et al.*, 2004). Despite the presence of the vacuolar Fe^2+^ and Mn^2+^ transporter CCC1 (Li *et al.*, 2001) in K667, the triple *Δpmc1Δvcx1Δcnb* deletion results in severe impairment of the Mn^2+^ homeostasis and in an increased sensitivity to Mn. As CsMTP6 restores the growth of K667 cells under high Mn conditions, it may be assumed that the Mn-sensitive phenotype of this strain results from the toxic effect of Mn on mitochondria. As shown in Fig. 6B, C, the Mn content and Mn-SOD activity were higher in the mitochondria of K667 when compared to the wild-type yeast. These results indicate that Mn-induced toxicity can increase the production of reactive oxygen species in the mitochondria of the K667 strain. Mn has already been shown to increase mitochondrial H_2_O_2_ production over a physiological as well as toxic range of concentrations in human neuroblastoma cells (Fernandes *et al.*, 2017). In addition, it has been shown in rat primary neuron cultures that toxic Mn concentrations negatively affect the mitochondrial membrane potential and the activity of complex II, and lead to DNA fragmentation that results in apoptotic-like neuronal death (Malecki, 2001). The accumulation of Mn in mitochondria and in mitochondria-rich tissues *in vivo* also directly interferes with oxidative phosphorylation, probably by binding to the F_1_-ATPase (Gavin *et al.*, 1992). Hence, the mechanism for Mn-induced toxicity is thought to result from Mn-induced oxidative damage, mitochondrial dysfunction, and the resultant apoptotic cell death (Gavin *et al.*, 1992; Malecki, 2001; Fernandes *et al.*, 2017). Therefore, we can assume that the CsMTP6-mediated Mn efflux from mitochondria and the subsequent CCC1-mediated Mn sequestration in the vacuole could protect the mitochondria of K667 cells from Mn toxicity, and thus render the strain more tolerant to excess Mn. In contrast, the CsMTP6-mediated Fe efflux from mitochondria could not protect Δ*ccc1* cells from excess Fe, as yeast lacking CCC1 are unable to accumulate excess Fe in the vacuole.

RETRACTED

In contrast to CsMTP6, the members of the Fe/Zn-CDF subgroup characterized so far, including bacterial FieF-like and WmFieF-like proteins and the fungal MMT-like transporters, are probably not capable of Mn transport (Li and Kaplan, 1997; Grünberg *et al.*, 2001; Grass *et al.*, 2005), suggesting functional diversification between the Fe/Zn-CDF transporters from different species. Interestingly, a phylogenomic analysis of CDF proteins from different organisms, including 56 newly identified CDF homologs, found 18 additional clades within the three substrate-specific groups Mn-CDF, Zn-CDF, and Fe/Zn-CDF that contain proteins with potentially new metal specificities (Mn, Fe, Co, Zn, Zn/Cd, Ni/Co) (Cubillas *et al.*, 2013). In this analysis, MTP6 as well as the MMT1 and MMT2 proteins were classified in clade II that contains the Fe-specific CDFs; however, this clade originates from the same ancestor as the neighboring clade I, containing the Mn-specific CDFs (Cubillas *et al.*, 2013). Hence, the broader specificity of MTP6 for Mn and Fe may be an ancient feature that has been retained in some members of clades 1 and 2. In addition, the novel Mn/Fe subfamily has recently been identified in clade VI of CDFs from α-proteobacteria (Cubillas *et al.*, 2014), supporting the hypothesis that some members of the CDF family are capable of transporting both Mn and Fe.

### *CsMTP6* expression affects mitochondrial Fe and Mn levels in Arabidopsis protoplasts

The similar patterns of CsMTP6 localization in plants and yeast suggested that CsMTP6 contributes to the export of Fe and Mn from the mitochondria of plant cells. To verify the functionality of the cucumber protein in plants, we determined the mitochondrial Fe and Mn contents in Arabidopsis protoplasts expressing *CsMTP6-GFP* that were pre-incubated with either 100 µM FeSO_4_-EDTA or 100 µM MnSO_4_ prior to preparation of the mitochondria. The presence of CsMTP6 in the isolated mitochondria was confirmed by western blotting (Fig. 7A). As shown in Fig. 7B, C, and Dataset S4 at Dryad, the Fe and Mn contents in mitochondria containing CsMTP6-GFP were approximately 2-fold lower when compared to mitochondria prepared from protoplasts transformed with an empty vector. In addition, CsMTP6 expression in the protoplasts resulted in a 30% decrease in Mn-SOD activity (Fig. 7D). These results confirmed the hypothesis that CsMTP6 is involved in the efflux of Fe and Mn from the mitochondria of plant cells. Although the direct involvement of CsMTP6 in Fe and Mn extrusion needs to be confirmed, it is not surprising that Mn would share the same transporter with Fe. Both metals are known to share the same plasma membrane uptake transport systems, including the IRT1 (Korshunova *et al.*, 1999), YSL2 (Koike *et al.*, 2004), and NRAMP1 transporters (Cailliatte *et al.*, 2010; Castaings *et al.*, 2016). In addition, Fe and Mn share the same tonoplast transporters involved in the vacuolar sequestration (VIT1 and MTP8) or remobilization (NRAMP3 and NRAMP4) of metal ions (Thomine *et al.*, 2003; Lanquar *et al.*, 2005, 2010; Chu *et al.*, 2017; Eroglu *et al.*, 2017). The broader specificity of metal transporters to both metals probably results from the similarity of the two ions: Mn is structurally and chemically similar to Fe due to comparable atomic radii and electron shells, which allows for similar reactions, transport, and trafficking mechanisms by substitution of Fe for Mn (Smith *et al.*, 2017). Therefore, we may assume that both metals can compete for transport by CsMTP6 and that the excess of one metal in the mitochondria should negatively affect the efflux of the other from the mitochondrial matrix. However, the biological relevance of this phenomenon remains to be determined.

RETRACTED

**Fig. 7.** Effects of *CsMTP6* expression on mitochondrial Fe and Mn contents and Mn-SOD activity in Arabidopsis protoplasts. (A) Western blot analysis of the purity of mitochondrial and plastidial fractions prepared from protoplasts expressing *CsMTP6* using primary antibodies raised against GFP (to detect CsMTP6-GFP), and marker proteins for plastids (Toc75) and mitochondria. The mitochondria and plastid fractions were prepared from protoplasts by discontinuous density gradient centrifugation in Percoll. (B) Fe and (C) Mn content in the mitochondrial fraction prepared from Arabidopsis protoplasts expressing *CsMTP6* or transformed with the empty vector. Data are means (±SD) from three separate experiments. (D) Mitochondrial Mn-SOD activity in protoplasts expressing *CsMTP6*. Data are means (±SD) from three separate experiments, expressed as enzyme units (U). Significant differences were determined using Student’s *t*-test.

The contribution of CsMTP6 to Fe and Mn export from the mitochondria suggests that plant MTP6 proteins may be involved in the protection of mitochondria from excess Fe and Mn and/or in the remobilization of both ions, particularly Fe, from mitochondria under deficiency. Similar to Fe, Mn is also required for the proper function of mitochondria, as a co-factor of the mitochondrial Mn-SOD, an enzyme involved in the protection of mitochondria from the harmful effects of superoxide radicals (Miller, 2012). However, excess Mn, like excess Fe, is toxic for mitochondria and therefore the levels of both must be tightly controlled, and MTP6 proteins could be involved in such control. In order to test this hypothesis, we further measured the transcript and protein levels of CsMTP6 under different Mn and Fe availability.

RETRACTED

### Root expression of *CsMTP6* varies with different Fe availability

The levels of *CsMTP6* transcript were significantly elevated both by Fe excess and by Fe deficiency, but there was no effect of different Mn availability (Fig. 8A, Dataset S1 at Dryad). Consistent with the results from the expression assay, the mitochondrial level of CsMTP6 was also increased under elevated Fe concentrations and Fe deficit but remained unchanged by different Mn treatments (Fig. 8B). These results indicate that CsMTP6 activity is regulated by Fe but not by Mn, and that the Fe-mediated increase in mitochondrial CsMTP6 content could be important for the maintenance of mitochondrial and cytosolic Fe homeostasis. Interestingly, the Arabidopsis vacuolar transporters NRAMP3 and NRAMP4 are also regulated by Fe but not Mn availability (Lanquar *et al.*, 2010), indicating that the response of plant cells to the two metals involves different signaling pathways.

**Fig. 8.** The levels of *CsMTP6* transcript and protein under different Fe and Mn availability. (A) Real-time analysis of *CsMTP6* expression in the roots of 2-week-old cucumber seedlings growing under control Fe (75 µM), control Mn (0.1 µM), excess Fe (1 mM), excess Mn (10 µM), Fe deficiency, or Mn deficiency. Data are mean *CsMTP6* transcript levels (±SD) relative to the constitutively expressed reference gene *CACS* calculated from the arithmetic means of Δ*C*p values obtained in three independent experiments. (B) Western blot analysis of CsMTP6 protein levels in mitochondria isolated from roots of cucumbers grown under different Fe and Mn treatments for 2 weeks. Immunoblots of the same mitochondria were probed with antibodies against mitochondrial COXII cytochrome oxidase to ensure equal loading of membrane protein (10 µg) onto SDS-PAGE. Significant differences were determined using Tukey’s test.

The enhanced CsMTP6-mediated efflux of Fe from the mitochondria can protect them from the toxic effects of an excess in conditions of Fe toxicity, or can supply the cellular metabolism with Fe in conditions of deficiency. Thus, our results support the current hypothesis on the possible function of plant mitochondria in Fe storage (Vigani *et al.*, 2013). It has previously been shown that mitochondria, similarly to plastids, are able to accumulate the Fe-storing protein ferritin, and mitochondrial ferritin has been discovered in Arabidopsis, pea, and cucumber (Zancani *et al.*, 2004; Tarantino *et al.*, 2010; Vigani *et al.*, 2013). The localization of ferritin in the mitochondria of cucumber roots indicated that root mitochondria are capable of storing Fe in a non-toxic form that can be remobilized by the cells in case of deficiency. We believe that plant MTP6 proteins are good candidates for the proteins involved in the remobilization of Fe from the mitochondrial pools in plant cells.

RETRACTED

To gain insights into the responses of the other Fe organellar transporters to different Fe availability, we have previously measured the root expression of genes encoding the cucumber homologs of Arabidopsis VIT1, MIT1, MIT2, ferroportin, and PIC1 (chloroplast iron permease) under Fe-deficient or -excess conditions (Migocka *et al.*, 2018*a*). In addition, we have studied the expression of another MTP protein of the Fe/Zn subgroup localized in the mitochondria, CsMTP7, and the expression of mitochondrial ferritin under the same conditions; in contrast to CsMTP6, CsMTP7 contributes to Fe loading into the mitochondria when expressed in yeast and Arabidopsis protoplasts (Migocka *et al.*, 2018*a*). Protein coding transcripts and protein levels of CsMTP7 and ferritin were significantly and rapidly increased upon exposure to a non-toxic elevated Fe concentration (500 µM), but were barely detected under Fe deficiency (Migocka *et al.*, 2018*a*). Hence, we assume that CsMTP7 and ferritin work in concert to increase the accumulation of Fe in plant mitochondria under elevated Fe conditions. These results confirm the hypothesis that, similar to plastids and the vacuole, mitochondria have also developed a high capacity for storing Fe. As CsMTP6 is involved in Mn/Fe efflux from mitochondria, we assume that plant MTP6 and MTP7 proteins might fulfil different physiological functions: taking into account the H^+^ gradient generated in the inner mitochondrial membrane, we may assume that CsMTP7 catalyses the import of Fe^2+^ into mitochondria via the symport mechanism, whereas CsMTP6 catalyses the export of Fe^2+^ and Mn^2+^ from mitochondria through a Fe^2+^(Mn^2+^)/H^+^ antiport (Migocka *et al.*, 2018*a*). Based on the effect of Fe on the expression of both proteins, we can hypothesize that CsMTP7 is up-regulated by elevated Fe to increase the mitochondrial content (for Fe storage), whereas CsMTP6 is up-regulated by elevated Fe to remove excess and reduce Fe toxicity, or by Fe deficiency to release Fe stored in mitochondria in order to meet cellular demands. Similar to CsMTP6, the vacuolar iron transporters NRAMP3 and NRAMP4 have been shown to be up-regulated under conditions of low Fe to release Fe stored in the vacuole to meet cellular demands during seed germination (Lanquar *et al.*, 2005). In addition to CsMTP7, iron mitoferrins mediate Fe transport into mitochondria. Nevertheless, both the cucumber genes encoding MITs are up-regulated upon Fe deficiency and are not affected by excess Fe (Migocka *et al.*, 2018*a*), suggesting that they may be crucial for the mitochondrial import of Fe under limiting conditions. The expression of other genes coding for proteins involved in Fe uptake and accumulation in cucumber roots is also altered only upon Fe deficiency (plasma membrane CsIRT1 and CsFRO2, CsIREG2/CsFNP2, chloroplast CsPIC1/CsTIC21) or is not affected by Fe availability (CsVIT1) (Migocka *et al.*, 2018*a*). These results suggest that mitochondrial Fe homeostasis is rapidly regulated by Fe excess and deficiency at the level of the transcription of *MIT*s, *MTP6*, and *MTP7*, whereas the accumulation of Fe in the plastids or vacuoles of cucumber roots is not altered following supplementation of Fe. Based on these results, we can conclude that the mitochondria of cucumber roots may play a very important role in maintaining cellular Fe homeostasis, and that the function of the other organellar Fe transporters in the roots may be predominantly related to the response of cucumber to Fe deficiency.

RETRACTED

In conclusion, this study supports the hypothesis that plant MTP6 proteins function in mitochondrial Mn/Fe efflux and can thus play an important role in the maintenance of mitochondrial and cytosolic Fe and Mn homeostasis. The mitochondrial localization and the Fe and Mn specificity of CsMTP6 provide novel insights into the functions of MTP proteins in plant cells.

## Data deposition

The following tables and figures are available at Dryad Data Repository: https://doi.org/10.5061/dryad.306sf0b, last accessed on October 19, 2018.

Table S1. Yeast strains used in this work.

Fig. S1. Organ expression pattern of *CsMTP6* in cucumber.

Fig. S2. ClustalW alignment of the *CsMTP6* nucleic acid and CsMTP6 amino acid sequences.

Fig. S3. Western blot analysis of mitochondria isolated from yeast expressing CsMTP6.

Fig. S4. Localization of CsMTP6 in Δ*zrc1*, K667, and Δ*smf1* cells.

Fig. S5. Effect of *CsMTP6* expression on yeast sensitivity to Zn, Ni, and Cd.

Dataset S1. *CsMTP6* expression data.

Dataset S2. Data for GDO activity in yeast.

Dataset S3. Data for metal content from mitochondria in yeast.

Dataset S4. Data for metal content in mitochondria of protoplasts.
